The article "Exploring the amino acid profile and microbial properties of locally sweet preserved kachra hareer (Terminalia chebula)" was retracted in 2024. Reasons: compromised peer review; unreliable results or conclusions; concerns about the peer review.

# Exploring the amino acid profile and microbial properties of locally sweet preserved kachra hareer (*Terminalia chebula*)

**DOI:** 10.1002/fsn3.2056

**Published:** 2020-12-13

**Authors:** Ali Ikram, Farhan Saeed, Haroon Munir, Muhammad Tauseef Sultan, Muhammad Afzaal, Aftab Ahmed, Faqir Muhammad Anjum

**Affiliations:** ^1^ Institute of Home and Food Sciences Government College University Faisalabad Pakistan; ^2^ Institute of Food Science and Nutrition Bahauddin Zakariya University Multan Pakistan; ^3^ The University of Gambia Serekunda Gambia

**Keywords:** amino acid profile, extractive values, hareer, mineral, vitamin C

## Abstract

The current research was designed to determine the amino acid profile and microbial properties of kachra hareer. For the purpose, kachra hareer was purchased with their brand names coded as S1, S2, S3, and S4 from five towns named as L1, L2, L3, L4, and L5. The samples were analyzed for their amino acid profile and microbial properties, while the water and alcohol extractive values were analyzed to obtain the different levels of purity during processing. The results explained that physicochemical analyses, that is, pH, moisture, acidity, and vitamin C, ranged from 4.67% to 9.44%, 22% to 40%, 0.054% to 1.44%, and 7.67% to 19.36%, respectively. However, essential amino acids histidine, isoleucine, leucine, methionine, phenylalanine, proline, threonine, and valine ranged from 470.3 to 484.5, 516.1 to 527.5, 805.5 to 817.4, 910.1 to 922.5, 240.2 to 250.5, 508.2 to 518.2, 1,160.5 to 1,172.6, 466.9 to 476.3, and 502.5 to 513.4 mg/kg, respectively, whereas nonessential amino acids alanine, arginine, aspartic acid cysteine, glutamic acid, serine, tyrosine, and glycine ranged from 612.7 to 628.2, 1,212.3 to 1,225.9, 7,254.2 to 7,258.8, ND, 1,561.2 to 1,575.2, 634.8 to 648.9, 618.4 to 630.4, and 712.8 to 723.7 mg/kg, respectively. Conclusively, sample S_2_ showed the maximum nutritional content and minimum microbial load.

## Graphical abstract

Different brands of sweet preserved hareer are checked for their microbial load. The nutritional profile of hareer was also checked.

## 1 INTRODUCTION

Hareer, a prudent tree used in traditional medications, goes to the family Combretaceae. It is generally called *Black myrobalan* or *Chebulic myrobalan*. The botanical name of hareer is *Terminalia chebula*. It is tremendously used in India, Asia, and Africa (Baliga et al., 2012); additionally, the herb has been widely used for the cure of diseases such as cancer, cardiovascular diseases, leprosy, ulcers, paralysis, arthritis, and gout. Further, the herb has been well stated to possess antidiabetic, antibacterial, antioxidant, antiviral, anticancer, antifungal, antimutagenic, antiulcer, and wound‐healing actions (Kannan et al., 2009).

Hareer is recognized to possess an extensive range of phytochemical ingredients. *Terminalia chebula* has several phytoconstituents such as tannins, amino acids, flavonoids, sterols, fixed oils, fructose, and resin. The main phytoconstituents in hareer are hydrolyzable tannins (which may differ from 32% to 34%) (Pathak et al., 2019). Tannin content differs with geographical variations.

It is productive in keeping the urease activity of *Helicobacter pylori* (*H. pylori*), an ever‐show bacterium worried in the improvement of ulcers, stomach malignancies, and gastritis (Singamaneni et al., 2020). Antibacterial activity of hareer against both Gram‐positive and Gram‐negative human pathogenic organisms has likewise been depicted (Akbar, 2020). It is compelling against the pathogenic yeast *dermatophytes* and *Epidermophyton*, *Floccosum*, *Candidaalbicans*, *Trichophyton rubrum*, and *Microsporum gypseum* (Vonshak et al., 2003). Its preventoria result in three dermatophytes (*Trichophyton* spp.) and three yeasts (*Candida* spp.) has likewise been recorded (Li et al., 2019).

The fruit of hareer provides 6.36 kJ/g of energy. Fruit contains protein (3.78%), carbohydrate (9.21%), and vitamin C (369 ppm), starch (1.22%), sucrose (3.74%), reducing sugars (7.56%), and reducing substances (11.5%). The weight of hareer fruit pulp is 2.99 g, fruit peel 0.40 g, and pit weight 1.51 g (Nigam et al., 2020).

## 2 MATERIALS AND METHODS

The present study was carried out in the Food Technology section and Postharvest section of Ayub Agriculture Research Institute Faisalabad (AARI).

### 2.1 Procurement of samples

The samples of sweet preserved hareer were procured from the towns of the local market of Pirmahal (L1), Toba Tek Singh (L2), Chiniot (L3), Janarawala (L4), and Faisalabad (L5). The flow line of the procedure for the sweetened preserved hareer included neutralization, presweeting, and post‐ or final sweetening using sucrose syrups both fresh and recycled ones. Samples of four well‐known brands (Latif, Yousaf, Khalid, and Aslam) of the product were taken randomly in triplicate from five different towns of the cities and were marked as S1, S2, S3, and S4 each, respectively.

### 2.2 Qualitative analyses

#### 2.2.1 Moisture

This test was performed to check the water content in sweet preserved hareer as described by the AACC (2000). An electric oven (WTE Binder Type B115 No. 86490) was used for moisture determination.

#### 2.2.2 Ash

Ash content was analyzed as described by AACC (2000) by using a weighing balance (GM 1501), analytical balance (Shimadzu ATX 224), and electric muffle furnace (Thermolyne 1400 Furnace).

#### 2.2.3 Acidity

Acidity was determined by the direct titration method as described by the AACC (2000).

#### 2.2.4 pH

This test was performed to determine the acidity or alkalinity as described by AACC (2000). In this case, pH meter (HI 2211 pH/ORP meter) was used.

#### 2.2.5 Vitamin C

Ascorbic acid was determined as described by the AACC (2000).

#### 2.2.6 Total soluble solids

This test was determined by the AOAC (1984) by using digital refractometer (HI 96801).

#### 2.2.7 Color

The color of sweet preserved hareer was determined by the AACC (2000). Digital reflectance colorimeter (color Tec‐PCM 3001378) was used.

#### 2.2.8 Extractive values

Extractive values are primarily useful for examining adulterated or exhausted drugs. The extractive values of the crude drug determine the quality and clarity of the drug. Thus, alcohol‐soluble and water‐soluble extractive values were determined by the specification number I.S. 1797‐1985 methods of test for species and condiments.

### 2.3 Microbial analysis

Hareer was tested for total plate count, *Salmonella*, and *E. coli* by the methods determined by AACC (2000).

### 2.4 Minerals

Fruit pulp was used for mineral analysis. The digestion method of Lierop (1976) was used for fruit sample preparations of Ca, K, P, and Mg, while Gorsuch (1959) for the preparations of Zn, Na, Fe, Cu, and Mn, Ca, Fe, Mn, Zn, Cu, and Mg were tested by using flame absorption, using a Varian Spectra AA‐30 Spectrophotometer and K and Na were measured by flame emission. Boron was tested by the quinalizarin method, P was determined by molybdovanado phosphoric acid method using a Technicon AutoAnalyzer II, and C1 was calculated by potentiometric technique AOAC (1984). S content was found by the MgNO3 method; Si by the gravimeter AOAC (1984); and Se by the diaminobenzidine reaction APHA (1979).

### 2.5 Amino acid analysis

For amino acid analysis, twenty to thirty mg of each sample was hydrolyzed for 23 hr in 4 ml of 6N HC1 under vacuum at 110°C and the hydrolysate was washed with distilled water through a glass wool column and brought to volume in a volumetric flask of 10 ml. The HCl from an aliquot of 0.5 ml was evaporated with KOH pellets in a desiccator, and the residue was taken up as an internal standard in 1 ml of pH 2.2 of the sodium citrate buffer (0.2 N) containing 250 nanomoles per ml of norleucine. To calibrate the analyzer, the Beckman amino acid standard for hydrolysate evaluation was used. The unit was a Beckman 121 MB Model, Beckman Instruments, Inc., Spinco Division, Palo Alto, California, fitted with a single column (2.8 mm bore × 300 mm in length) packed to a height of 210 mm with spherical resin exchange type AA‐10 Beckman. Another place was outlined in detail the chromatographic conditions used in these studies (Moore et al., 1958).

## 3 RESULTS AND DISCUSSION

The standard fruit (raw) was studied for parameters such as pH, moisture, ash, acidity, vitamin C, total soluble solids (TSS), color, minerals, and essential and nonessential amino acids.

### 3.1 Physicochemical analysis of processed hareer

Mean values regarding moisture content of sweet preserved hareer are given in Table 1, which indicated significant results. Results showed that the moisture content of sweet preserved hareer (control) is 39%. Moreover, the moisture content of different hareer (sweet preserved) samples ranged from 26% to 38%. The minimum value (26%) of moisture content has been found in the sample S3L1, which indicated the presence of greater TSS, while the maximum value (38%) was exhibited in S2L1. Results were also compared with Kumar et al. (2017) who observed the moisture content in hareer not less than 10%.

**TABLE 1:** Physicochemical analysis of sweet preserved hareer

Brand	Cities	Vit. C	pH	Moisture	Ash	TSS	Acidity	Color		
								*L*	*a*	*b*
Control		17.45 ± 0.39	9.67 ± 0.2	39 ± 0.43	0.97 ± 0.13	70.26 ± 0.21	0.2076 ± 0.1	39.86 ± 0.39	0.03 ± 0.02	−4.85 ± 0.14
S_1_	L_1_	10.45 ± 0.38	6.5 ± 0.4	35 ± 0.54	0.63 ± 0.35	63.43 ± 0.41	0.41 ± 0.39	34.87 ± 0.1	−2.48 ± 0.2	1.6 ± 0.3
	L_2_	11.61 ± 0.33	7.53 ± 0.35	26 ± 0.64	0.716 ± 0.27	60.26 ± 0.4	0.56 ± 0.38	33.10 ± 0.47	−2.45 ± 0.39	−1.52 ± 0.32
	L^3^	8.46 ± 0.36	7.58 ± 0.37	31 ± 0.3	0.69 ± 0.27	62.37 ± 0.5	0.386 ± 0.42	36.48 ± 0.3	0.45 ± 0.38	0.59 ± 0.37
	L_4_	7.57 ± 0.35	5.5 ± 0.3	29 ± 0.56	0.46 ± 0.3	58.54 ± 0.4	0.647 ± 0.05	32.44 ± 0.3	−3.39 ± 0.5	0.13 ± 0.03
	L_5_	11.67 ± 0.2	7 ± 0.95	32 ± 0.64	0.74 ± 0.1	57.2 ± 0.1	0.48 ± 0.08	31.55 ± 0.4	1.64 ± 0.4	0.59 ± 0.3
S_2_	L_1_	11.58 ± 0.37	8.46 ± 0.28	38 ± 0.65	0.84 ± 0.39	67.6 ± 0.41	0.186 ± 0.03	36.61 ± 0.37	−4.57 ± 0.3	−2.56 ± 0.2
	L_2_	9.63 ± 0.32	9.2 ± 0.3	34 ± 0.73	0.77 ± 0.2	66.5 ± 0.3	0.31 ± 0.33	38.53 ± 0.2	−1.67 ± 0.28	1.69 ± 0.3
	L^3^	16.74 ± 0.3	7.1 ± 0.4	35 ± 0.63	0.88 ± 0.1	66.6 ± 0.2	0.52 ± 0.37	37.7 ± 0.2	−3.54 ± 0.43	−2.07 ± 0.03
	L_4_	11.69 ± 0.14	8.53 ± 0.37	37 ± 0.75	0.78 ± 0.16	64.8 ± 0.1	0.054 ± 0.01	35.52 ± 0.3	−2.56 ± 0.3	−5.62 ± 0.42
	L_5_	15.74 ± 0.31	7.6 ± 0.3	32 ± 0.85	0.612 ± 0.23	69 ± 0.93	0.53 ± 0.4	36.44 ± 0.3	1.5 ± 0.42	0.67 ± 0.37
S_3_	L_1_	9.67 ± 0.38	5.7 ± 0.43	26 ± 0.74	0.52 ± 0.2	62.5 ± 0.4	0.59 ± 0.24	33.5 ± 0.3	2.09 ± 0.05	−3.69 ± 0.16
	L_2_	7.67 ± 0.2	6.44 ± 0.3	30 ± 0.74	0.64 ± 0.12	59.5 ± 0.2	0.42 ± 0.44	30.6 ± 0.41	−7.79 ± 0.12	0.05 ± 0.02
	L^3^	11.68 ± 0.25	7.4 ± 0.26	32 ± 0.93	0.53 ± 0.22	60 ± 0.94	0.318 ± 0.43	33.54 ± 0.37	−1.65 ± 0.17	−5.33 ± 0.3
	L_4_	7.74 ± 0.1	7.6 ± 0.1	27 ± 0.83	0.64 ± 0.27	61.6 ± 0.3	0.321 ± 0.27	35.47 ± 0.47	−7.5 ± 0.2	2.48 ± 0.32
	L_5_	7.36 ± 0.15	6.5 ± 0.1	29 ± 0.73	0.69 ± 0.21	58.4 ± 0.32	0.466 ± 0.3	36.08 ± 0.01	−6.64 ± 0.25	−3.77 ± 0.15
S_4_	L_1_	10.63 ± 0.2	7.44 ± 0.25	25 ± 0.93	0.56 ± 0.17	61.44 ± 0.3	0.51 ± 0.42	34.67 ± 0.25	−14.6 ± 0.41	2.87 ± 0.05
	L_2_	8.73 ± 0.2	5.44 ± 0.35	27 ± 0.8	0.67 ± 0.16	60.56 ± 0.35	0.43 ± 0.4	35.5 ± 0.42	−2.57 ± 0.27	4.59 ± 0.27
	L^3^	9.67 ± 0.3	7.6 ± 0.3	27 ± 0.4	0.42 ± 0.32	58.46 ± 0.35	0.44 ± 0.37	33.66 ± 0.27	−2.5 ± 0.21	−4.07 ± 0.02
	L_4_	6.72 ± 0.3	4.67 ± 0.2	33 ± 0.83	0.64 ± 0.2	57.47 ± 0.32	0.7 ± 0.3	35.47 ± 0.3	0.7 ± 0.14	3.57 ± 0.2
	L_5_	7.55 ± 0.13	6.56 ± 0.2	30 ± 0.2	0.84 ± 0.06	55.46 ± 0.37	0.21 ± 0.09	30.25 ± 0.15	3.6 ± 0.49	−11 ± 0.44

Mean values regarding the pH of sweet preserved hareer are given in Table 1, which indicated significant results. Results showed that the pH of hareer (control) is 9.67. Moreover, the pH of different hareer (sweet preserved) samples ranged from 4.67 to 9.2. The minimum acidic value (4.67) of pH has been found in sample S4L4, whereas the samples S1L4, S2L3, S3L1, S3L2, and S4L2, and S4L4 showed lower pH values because they were not neutralized properly and a little acidic nature was observed in those samples. Jirankalgikar et al. (2012) reported the acidic nature of the hareer having a pH value was 4. Mean values regarding ash content of sweet preserved hareer are given in Table 1, which indicated significant results. Results showed that the ash content of sweet preserved hareer (control) is 0.97%. Moreover, ash of different hareer (sweet preserved) samples ranged from 0.42% to 0.88%. The minimum value (0.42%) of ash content has been found in sample S4L3, while the maximum value (2.88%) was exhibited in S2L3. Keshava (2014) also noticed similar results and observed that the ash value in raw hareer fruit was 2.95%. Similar results were also given by Jirankalgikar et al. (2012). Mean values regarding the acidity of sweet preserved hareer are given in Table 1, which indicated significant results. Results showed that the acidity content of sweet preserved hareer (control) is 0.207%. Moreover, the acidity of different hareer (sweet preserved) samples ranged from 0.054% to 0.7%. The minimum value (0.054%) of ash content has been found in sample S2L4, while the maximum value (0.7%) was exhibited in S4L4. Higher values for acidity showed retention of acids during processing and relatively lesser neutralization of acids. The product became more palatable when properly neutralized, so it is considered a desirable feature for sweet preserved hareer fruit.

Mean values regarding vitamin C of sweet preserved hareer are given in Table 1, which indicated significant results. Results showed that the vitamin C content of sweet preserved hareer (control) is 17.45%. Moreover, vitamin C of different hareer (sweet preserved) samples ranged from 6.72% to 16.74%. The minimum value (6.72%) of vitamin C content has been found in sample S4L4, while the maximum value (16.74%) was exhibited in S2L3.

Mean values regarding TSS of sweet preserved hareer are given in Table 1, which indicated significant results. Results showed that the TSS content of sweet preserved hareer (control) is 64.26%. Moreover, TSS of different hareer (sweet preserved) samples ranged from 56% to 71%. The minimum value (56%) of TSS content has been found in sample S2L5, while the maximum value (71%) was exhibited in S1L3.

Mean values regarding the color of sweet preserved hareer are given in Table 1, which indicated significant results. Results showed that the color of sweet preserved hareer (control) is “*L*” 39.86, “*a*” 0.03, and “*b*” −4.85. Moreover, the color of different hareer (sweet preserved) samples ranged from 30.25 to 38.53 in “*L*”, −7.79 to 3.6 in “*a*,” and −11 to 4.59 in all the fruit samples. “***L***” values were observed maximum positively in S1L3, S2L1, S2L2, and S3L5 as 36.48, 36.61, 38.53, and 36.08, respectively. The highest value of “*L*” showed that the product is given additional colors while processing. Higher values for positive “***a***” were found in S3L1 and S4L5 as 2.09 and 3.6, respectively, which explored the natural reddish tinge of fruit. Moreover, negative value was observed in S3L2 as −7.79, which showed the presence of green color due to the use of additional colorings. “***b***” values were found positive in S4L4 and S4L2 as 3.57 and 4.59, respectively. The maximum negative “*b*” value was found in S4L5 as −11.

Mean values regarding water‐soluble and alcohol‐soluble extractive values of sweet preserved hareer are given in Table 2, which indicated significant results. Results showed that the water‐soluble extractive values and alcohol‐soluble extractive values of sweet preserved hareer (control) are 65% and 60%, respectively. Water‐soluble extractive value ranged from 47% to 64%, whereas the alcohol‐soluble extractive value ranged from 37% to 59% in all the sweet preserved samples. The maximum water‐soluble extractive value (64%) was observed in S2L3. Meanwhile, the minimum water‐soluble extractive value (47%) was observed in S3L3. A higher alcohol‐soluble extractive value (59%) was observed in S2L3. A minimum alcohol‐soluble extractive value (37%) was observed in S4L2. Higher extractive values in certain samples showed inadvertent use of freshly prepared sugar solutions for preservation. The results showing the lower water‐ and alcohol‐soluble extractive values generally depicted the story of using recycled sugar solutions without having a standard concentration.

**TABLE 2:** Extractive values of sweet preserved hareer

Brands	Cities	Water‐soluble extractive value	Alcohol‐soluble extractive value
Control		65 ± 0.54	60 ± 0.87
S_1_	L_1_	57 ± 0.32	41 ± 0.44
	L_2_	52 ± 0.23	56 ± 0.99
	L^3^	52 ± 0.62	55 ± 0.64
	L_4_	58 ± 0.63	58 ± 0.84
	L_5_	55 ± 0.42	57 ± 0.85
S_2_	L_1_	60 ± 0.64	58 ± 0.94
	L_2_	62 ± 0.92	57 ± 0.49
	L^3^	64 ± 0.53	59 ± 0.84
	L_4_	61 ± 0.72	56 ± 0.84
	L_5_	63 ± 0.23	55 ± 0.84
S_3_	L_1_	60 ± 0.56	53 ± 0.74
	L_2_	48 ± 0.64	49 ± 0.85
	L^3^	47 ± 0.64	47 ± 0.83
	L_4_	61 ± 0.66	39 ± 0.95
	L_5_	53 ± 0.75	47 ± 0.94
S_4_	L_1_	57 ± 0.93	42 ± 0.9
	L_2_	52 ± 0.85	37 ± 0.3
	L^3^	58 ± 0.74	56 ± 0.5
	L_4_	53 ± 0.84	51 ± 0.3
	L_5_	58 ± 0.83	53 ± 0.4

### 3.2 Microbial analysis of processed hareer

#### 3.2.1 Total plate count

Mean values regarding TPC of sweet preserved hareer are given in Table 3, which indicated significant results. Results showed that the TPC of sweet preserved hareer (control) is 5.88 × 10^6^ CFU/g. Moreover, the TPC of different hareer (sweet preserved) samples ranged from 3.06 × 10^6^ to 8.54 × 10^6^ CFU/g. The minimum load of microbes (3.06 × 10^6^) has been found in sample S2L2, while the maximum load of microbes (8.54 × 10^6^) was exhibited in S3L3. The samples were tested for their food safety point of view and observed that the microorganisms (*salmonella* and *E. coli*) are dangerous for human health as nil. Hareer showed itself antimicrobial properties. Kim et al. (2006) studied the extract of *T. chebula* fruit, and some biologically active components were isolated and tested against *Salmonella* and *Escherichia coli*. The strong and moderate inhibitory activity was observed against those microorganisms.

**TABLE 3:** Microbial analysis of sweet preserved hareer

Brands	Cities	TPC	*E. coli*	*Salmonella*
Control		5.88 × 10^6^ ± 0.03	ND	ND
S_1_	L_1_	4 × 10^6^ ± 0.2	ND	ND
	L_2_	5.49 × 10^6^ ± 0.34	ND	ND
	L^3^	6.70 × 10^6^ ± 0.2	ND	ND
	L_4_	8 × 10^6^ ± 0.2	ND	ND
	L_5_	8.32 × 10^6^ ± 0.02	ND	ND
S_2_	L_1_	5.71 × 10^6^ ± 0.08	ND	ND
	L_2_	3.06 × 10^6^ ± 0.11	ND	ND
	L^3^	5.88 × 10^6^ ± 0.07	ND	ND
	L_4_	4.41 × 10^6^ ± 0.03	ND	ND
	L_5_	6.4 × 10^6^ ± 0.04	ND	ND
S_3_	L_1_	7.4 × 10^6^ ± 0.2	ND	ND
	L_2_	7 × 10^6^ ± 0.2	ND	ND
	L^3^	8.54 × 10^6^ ± 0.05	ND	ND
	L_4_	8.4 × 10^6^ ± 0.1	ND	ND
	L_5_	7.03 × 10^6^ ± 0.02	ND	ND
S_4_	L_1_	6.4 × 10^6^ ± 0.2	ND	ND
	L_2_	5.4 × 10^6^ ± 0.05	ND	ND
	L^3^	4.8 × 10^6^ ± 0.02	ND	ND
	L_4_	8 × 10^6^ ± 0.2	ND	ND
	L_5_	4.9 × 10^6^ ± 0.1	ND	ND

#### 3.2.2 Minerals

Mean values regarding mineral content of sweet preserved hareer are given in Table 4, which indicated significant results. Results showed that the phosphorus content of different samples ranged from 640.4 to 654.2 mg/kg; moreover, the phosphorus content of sweet preserved hareer (control) is 656 mg/kg. The minimum value of phosphorus content has been found in sample S4L5, while the maximum value was exhibited in S2L1. The potassium content of different sweet preserved hareer samples ranged from 9,678.3 to 9,691.1 mg/kg; moreover, the potassium content of sweet preserved hareer (control) is 9,692 mg/kg. The minimum value of potassium content has been found in sample S4L5, while the maximum value was exhibited in S2L3. The calcium content of different sweet preserved hareer samples ranged from 1,278.2 to 1,290.6 mg/kg; moreover, the calcium content of sweet preserved hareer (control) is 1,291.6 mg/kg. The minimum value of calcium content has been found in sample S3L3, while the maximum value was exhibited in S2L3. The magnesium content of different sweet preserved hareer samples ranged from 669.5 to 681.6 mg/kg; moreover, the magnesium content of sweet preserved hareer (control) is 682.6 mg/kg. The minimum value of magnesium content has been found in sample S1L3, while the maximum value was exhibited in S2L5. The sulfur content of different sweet preserved hareer samples ranged from 668.4 to 679.6 mg/kg; moreover, the sulfur content of sweet preserved hareer (control) is 679.05 mg/kg. The minimum value of sulfur content has been found in sample S1L1, whereas the maximum value was exhibited in S2L3. The iron content of different sweet preserved hareer samples ranged from 28.6 to 39.5 mg/kg; furthermore, the iron content of sweet preserved hareer (control) is 40.4 mg/kg. The minimum value of iron content has been found in sample S4L4, while the maximum value was exhibited in S2L3.

**TABLE 4:** Minerals analyses of sweet preserved hareer

Brand	Cities	Phosphorous mg/kg	Potassium mg/kg	Calcium mg/kg	Magnesium mg/kg	Sulfur mg/kg	Iron mg/kg	Manganese mg/kg	Zinc mg/kg	Boron mg/kg	Copper mg/kg	Sodium mg/kg	Chloride mg/kg	Selenium mg/kg	Silica mg/kg
Control		656 ± 1.3	9,692.1 ± 0.7	1,291.6 ± 1	682.6 ± 1.2	679.05 ± 3	40.4 ± 0.7	18.2 ± 0.4	45.5 ± 0.7	43.1 ± 0.5	15.4 ± 0.6	78.4 ± 0.6	1,428 ± 0.5	11.8 ± 0.6	555.6 ± 0.2
S_1_	L_1_	649.3 ± 0.7	9,682.2 ± 0.4	1,286.4 ± 1	672.2 ± 0.8	668.4 ± 0.9	30.2 ± 0.8	8.3 ± 0.7	34.9 ± 0.5	33.4 ± 0.6	5.73 ± 0.5	69.8 ± 0.4	1,421 ± 0.6	4.8 ± 0.7	547.5 ± 0.3
	L_2_	647.4 ± 1	9,685.2 ± 0.3	1,281.5 ± 0.9	674.4 ± 0.9	671.3 ± 0.7	34.6 ± 0.8	6.2 ± 0.7	35.7 ± 0.9	32.9 ± 0.3	7.5 ± 0.7	65.0 ± 0.8	1,418.6 ± 0.7	3.8 ± 0.5	545 ± 1.4
	L^3^	643.6 ± 0.9	9,680.6 ± 0.6	1,284.6 ± 1	669.5 ± 0.7	674.5 ± 1	32.6 ± 0.8	10.1 ± 0.8	32.3 ± 0.8	35.4 ± 0.6	4.4 ± 0.7	68.2 ± 0.6	1,416.7 ± 0.9	1.7 ± 0.6	542.9 ± 0.7
	L_4_	646.5 ± 1	9,681.2 ± 0.6	1,280.5 ± 1	670.7 ± 0.8	670.3 ± 1	28.7 ± 1	7.4 ± 0.7	31.46 ± 0.5	30.56 ± 0.5	6.4 ± 0.6	66.1 ± 0.5	1,419.4 ± 1	5.8 ± 0.5	546.8 ± 0.7
	L_5_	645.7 ± 0.4	9,684.2 ± 0.8	1,283.7 ± 1	671.8 ± 0.7	672.2 ± 0.7	29.2 ± 1	9.4 ± 0.7	36.2 ± 0.8	31.4 ± 0.7	8.4 ± 0.8	70.2 ± 0.6	1,420.3 ± 0.4	6.9 ± 0.5	544.8 ± 0.7
S_2_	L_1_	654.2 ± 1	9,690.7 ± 0.4	1,288.9 ± 1	680.7 ± 1	676.5 ± 0.8	38.5 ± 0.7	16.3 ± 0.7	43.5 ± 0.6	41.4 ± 0.6	14.6 ± 0.6	76.7 ± 0.7	1,426.7 ± 1	10.7 ± 0.5	554.8 ± 0.7
	L_2_	652.4 ± 0.6	9,688.9 ± 0.7	1,289.3 ± 0.9	678.6 ± 1	678.5 ± 0.8	36.5 ± 0.6	14.9 ± 0.6	45.2 ± 0.7	40.8 ± 0.7	12.06 ± 0.6	74.3 ± 0.9	1,425.5 ± 0.7	9.9 ± 0.5	552.4 ± 0.8
	L^3^	650.1 ± 0.9	9,691.1 ± 0.6	1,290.6 ± 1	676.6 ± 1	679.6 ± 1	39.5 ± 0.8	15.4 ± 0.7	42.3 ± 0.5	39.5 ± 0.6	9.3 ± 0.7	71.6 ± 0.6	1,423.2 ± 0.9	7.7 ± 0.7	551.9 ± 0.7
	L_4_	651.8 ± 0.7	9,687.06 ± 0.4	1,286.6 ± 1	679.5 ± 1	677.2 ± 0.8	35.3 ± 0.7	14.3 ± 0.5	44.1 ± 0.6	37 ± 0.5	13.2 ± 0.6	73.5 ± 0.5	1,427.1 ± 0.4	6.7 ± 0.5	550.5 ± 0.2
	L_5_	653.4 ± 0.8	9,686.2 ± 0.7	1,285.7 ± 1	681.6 ± 0.9	675.3 ± 1	37.1 ± 0.7	11.2 ± 0.6	40.6 ± 0.6	42.3 ± 0.6	10.06 ± 0.6	77.4 ± 0.6	1,422.6 ± 0.4	11.5 ± 0.6	548.8 ± 0.8
S_3_	L_1_	648.2 ± 0.5	9,682.7 ± 0.7	1,281.2 ± 1	673.6 ± 1	675.5 ± 0.8	33.4 ± 0.8	10.3 ± 0.7	35.2 ± 0.6	33.3 ± 0.6	5.3 ± 0.5	69.03 ± 0.8	1,419.4 ± 0.6	6.8 ± 0.5	545.8 ± 0.7
	L_2_	645.8 ± 0.9	9,684.3 ± 0.5	1,280.4 ± 1	671.7 ± 1	670.9 ± 1	30.1 ± 0.7	8.4 ± 0.5	37.2 ± 0.7	33.5 ± 0.7	7.7 ± 0.6	68.5 ± 0.6	1,418.4 ± 0.6	4.4 ± 0.4	543.4 ± 0.9
	L^3^	646.4 ± 0.9	9,680.7 ± 0.5	1,278.2 ± 0.7	675.7 ± 1	669.1 ± 0.8	31.4 ± 0.7	6.5 ± 0.5	39.4 ± 0.6	33.1 ± 0.7	4.4 ± 0.6	67.1 ± 0.8	1,420.2 ± 0.8	5.7 ± 0.5	540.3 ± 0.9
	L_4_	643.5 ± 0.7	9,683.2 ± 0.8	1,283.8 ± 0.7	674.5 ± 0.7	673.5 ± 0.8	29.5 ± 0.7	9.4 ± 0.5	34.2 ± 0.8	33.2 ± 0.8	6.4 ± 0.5	65.5 ± 0.6	1,416.2 ± 0.7	1.6 ± 0.4	546.1 ± 0.5
	L_5_	647.3 ± 0.4	9,685.3 ± 0.7	1,282 ± 1	670.7 ± 1	671.7 ± 0.6	30.9 ± 0.8	7.2 ± 0.7	35.8 ± 0.4	33.3 ± 0.5	3.5 ± 0.6	70.5 ± 0.7	1,415.6 ± 0.7	3.8 ± 0.5	542.1 ± 0.5
S_4_	L_1_	646.7 ± 0.3	9,684.3 ± 0.7	1,285 ± 1	673.6 ± 0.3	674.2±	33.7 ± 0.9	8.4 ± 0.8	37.2 ± 0.7	35.5 ± 0.6	6.6 ± 0.7	68 ± 0.6	1,418.4 ± 0.5	5.9 ± 0.6	546.3 ± 0.5
	L_2_	641.6 ± 0.5	9,681.2 ± 0.5	1,284.7 ± 0.7	673.6 ± 1	669.3 ± 1	30.5 ± 06	6.1 ± 0.6	35.9 ± 0.7	33.6 ± 0.5	5.2 ± 0.4	63.6 ± 0.5	1,419.3 ± 0.4	2.7 ± 0.6	545.2 ± 0.6
	L^3^	643.4 ± 0.4	9,682.1 ± 0.6	1,282.5 ± 1	673.5 ± 1	672.2 ± 0.7	31.6 ± 0.7	5.3 ± 0.6	32.3 ± 0.6	30.03 ± 0.7	3.8 ± 0.5	65.3 ± 0.4	1,413.3 ± 0.5	1.7 ± 0.5	544.9 ± 0.6
	L_4_	645.7 ± 0.4	9,680.7 ± 0.3	1,278.5 ± 1	673.6 ± 0.9	670.8 ± 0.7	28.6 ± 1	9.06 ± 0.5	34.2 ± 0.6	28.5 ± 0.5	2.6 ± 0.5	67.2 ± 0.8	1,415.3 ± 0.9	4.7 ± 0.5	541.2 ± 0.6
	L_5_	640.7 ± 0.4	9,678.3 ± 0.5	1,280.9 ± 0.7	673.5 ± 1	671.1 ± 0.6	29.1 ± 0.6	10.3 ± 0.7	33.6 ± 0.5	31.2 ± 1	8.1 ± 0.8	69.1 ± 0.7	1,417.4 ± 0.6	5.7 ± 0.5	543.2 ± 0.5

The manganese content of different sweet preserved hareer samples ranged from 5.3 to 16.3 mg/kg; moreover, the manganese content of sweet preserved hareer (control) is 18.2 mg/kg. The minimum value of manganese content has been found in sample S4L3; however, the maximum value was exhibited in S2L1. The zinc content of different sweet preserved hareer samples ranged from 31.46 to 45.2 mg/kg. Moreover, the zinc content of sweet preserved hareer (control) is 45.5 mg/kg. The minimum value of zinc content has been found in sample S1L4, while the maximum value was exhibited in S2L2. The boron content of different sweet preserved hareer samples ranged from 28.5 to 42.3 mg/kg; moreover, the boron content of sweet preserved hareer (control) is 43.1 mg/kg. The minimum value of boron content has been found in sample S4L4, while the maximum value was exhibited in S2L5. The copper content of different sweet preserved hareer samples ranged from 3.5 to 14.6 mg/kg; moreover, the copper content of sweet preserved hareer (control) is 15.4 mg/kg. The minimum value of copper content has been found in sample S3L5, while the maximum value was exhibited in S2L1. The copper content of different sweet preserved hareer samples ranged from 63.6 to 77.4 mg/kg; moreover, the copper content of sweet preserved hareer (control) is 78.4 mg/kg. The minimum value of copper content has been found in sample S4L2, whereas the maximum value was exhibited in S2L5.

The chloride content of different sweet preserved hareer samples ranged from 1,413.3 to 1,427.1 mg/kg; moreover, the chloride content of sweet preserved hareer (control) is 1,428 mg/kg. The minimum value of chloride content has been found in sample S4L3, while the maximum value was exhibited in S2L4. Selenium content of different sweet preserved hareer samples ranged from 1.6 to 11.5 mg/kg; moreover, the selenium content of sweet preserved hareer (control) is 11.8 mg/kg. The minimum value of selenium content has been found in sample S3L4, while the maximum value was exhibited in S2L5. The silica content of different sweet preserved hareer samples ranged from 540.3 to 554.8 mg/kg; moreover, the silica content of sweet preserved hareer (control) is 555.6 mg/kg. The minimum value of silica content has been found in sample S3L3, while the maximum value was exhibited in S2L1. Similar results were also examined by Barthakur and Arnold (1991).

#### 3.2.3 Essential amino acid

Mean values regarding essential amino acid content of sweet preserved hareer are given in Table 5, which indicated significant results. Results showed that the histidine content of different sweet preserved hareer samples ranged from 470.3 to 484.5 mg/kg; moreover, the histidine content of sweet preserved hareer (control) is 485 mg/kg. The minimum value of histidine content has been found in sample S3L4, while the maximum value was exhibited in S2L2. Isoleucine content of different sweet preserved hareer samples ranged from 516.1 to 527.5 mg/kg; moreover, the isoleucine content of sweet preserved hareer (control) is 529.8 mg/kg. The minimum value of isoleucine content has been found in sample S4L1, while the maximum value was exhibited in S2L2. The leucine content of different sweet preserved hareer samples ranged from 805.5 to 817.4 mg/kg; moreover, the leucine content of sweet preserved hareer (control) is 818.3 mg/kg. The minimum value of leucine content has been found in sample S4L3, while the maximum value was exhibited in S2L3.

**TABLE 5:** Essential amino acid profile of sweet preserved hareer

Brand	Cities	Histidine mg/kg	Isoleucine mg/kg	Lucien mg/kg	Lysine mg/kg	Methionine mg/kg	Phenylalanine mg/kg	Proline mg/kg	Threonine mg/kg	Valine mg/kg
Control		485 ± 0.55	529.8 ± 0.75	818.3 ± 1	923.43 ± 0.66	251.43 ± 0.95	520.53 ± 0.75	1,173.13 ± 0.7	478.2 ± 0.81	514.8 ± 0.55
S_1_	L_1_	474.8 ± 0.55	521.4 ± 1.05	810.5 ± 1.2	916.4 ± 0.7	246.7 ± 0.98	513.36 ± 0.85	1,166.6 ± 0.86	468.13 ± 0.86	507.7 ± 1.05
	L_2_	476.2 ± 0.7	519.6 ± 0.6	806.5 ± 0.85	913.9 ± 0.5	244.3 ± 0.5	510.3 ± 1.1	1,162.4 ± 0.9	471.36 ± 0.75	504.4 ± 0.65
	L^3^	479.2 ± 0.76	522.83 ± 0.75	807.6 ± 0.8	911.03 ± 0.8	241.6 ± 0.8	508.2 ± 0.7	1,163.5 ± 0.8	467.8 ± 0.65	503.5 ± 53
	L_4_	474.8 ± 0.6	517.6 ± 0.95	809.4 ± 1.05	912.1 ± 0.75	238.4 ± 1.05	511.2 ± 0.6	1,161.5 ± 0.75	469.56 ± 0.75	502.56 ± 0.7
	L_5_	473.3 ± 0.6	516.4 ± 0.80	808.4 ± 1.15	910.1 ± 0.7	240.9 ± 0.8	517.1 ± 13	1,160.5 ± 0.75	466.9 ± 0.85	506.1 ± 0.8
S_2_	L_1_	479.8 ± 0.6	524.4 ± 0.8	816.55 ± 1.07	921.6 ± 0.85	249.5 ± 0.95	518.2 ± 0.7	1,169.5 ± 0.8	476.3 ± 0.5	512.3 ± 0.75
	L_2_	484.5 ± 0.6	527.5 ± 0.8	814.6 ± 1.13	922.5 ± 1.15	246.2 ± 0.65	516.6 ± 0.76	1,172.6 ± 0.9	472.5 ± 0.9	509.53 ± 0.9
	L^3^	482.83 ± 0.6	525.5 ± 0.7	817.4 ± 0.7	919.5 ± 1.15	247.6 ± 0.8	513.1 ± 0.8	1,168.7 ± 0.8	475.4 ± 0.9	507.6 ± 1.15
	L_4_	480.1 ± 0.6	524.5 ± 0.7	814.4 ± 0.9	917.5 ± 0.8	245.5 ± 0.8	515.1 ± 0.75	1,170.5 ± 1.25	469.3 ± 0.8	511.7 ± 0.6
	L_5_	478.8 ± 0.6	523.7 ± 0.6	813.6 ± 0.7	920.6 ± 0.8	250.5 ± 0.9	514.1 ± 0.65	1,169.6 ± 0.75	474.4 ± 0.8	513.4 ± 0.6
S_3_	L_1_	478.2 ± 0.5	521.8 ± 0.6	810.3 ± 0.96	918.2 ± 0.9	247.2 ± 0.6	515.7 ± 0.5	1,168.6 ± 1.25	469.2 ± 0.8	508.5 ± 0.7
	L_2_	476.9 ± 0.6	520.3 ± 0.8	812.4 ± 0.9	917.5 ± 0.8	244.2 ± 0.65	513.2 ± 0.6	1,165.3 ± 0.8	468.6 ± 0.9	510.5 ± 0.7
	L^3^	472.8 ± 0.5	517.5 ± 0.7	806.6 ± 1.19	919.8 ± 0.5	241.5 ± 0.8	510.2 ± 0.65	1,163.3 ± 1.05	474.4 ± 1.04	505.5 ± 1.01
	L_4_	470.3 ± 0.5	516.8 ± 0.7	807.4 ± 0.8	914.6 ± 1.2	238.3 ± 0.75	509.5 ± 0.7	1,160.5 ± 0.8	471.8 ± 0.9	507.6 ± 0.7
	L_5_	473.7 ± 0.7	519.8 ± 0.6	808.5 ± 0.8	910.4 ± 1.05	240.2 ± 0.6	511.4 ± 0.7	1,162.03 ± 0.7	470.5 ± 0.6	503.3 ± 1.06
S_4_	L_1_	474.6 ± 0.4	516.1 ± 0.6	809.2 ± 0.9	917.4 ± 1.01	245 ± 0.7	514.2 ± 0.7	1,166.4 ± 0.8	467.6 ± 0.7	508.06 ± 0.7
	L_2_	478.6 ± 0.5	522.6 ± 0.8	810.8 ± 0.3	916.4 ± 1.1	243.7 ± 1.08	512.9 ± 0.6	1,164.5 ± 0.7	469.3 ± 0.6	503.1 ± 0.8
	L^3^	476.8 ± 0.5	517.5 ± 0.7	805.5 ± 0.8	913.5 ± 1.2	241.4 ± 1	508.9 ± 0.8	1,161.6 ± 0.8	472.5 ± 0.8	507.8 ± 0.65
	L_4_	479.2 ± 0.6	520.4 ± 0.8	811.3 ± 0.7	912.3 ± 0.9	240.3 ± 0.7	510.7 ± 0.8	1,160.8 ± 1.05	474.1 ± 0.8	506.2 ± 0.6
	L_5_	472.6 ± 0.3	523.7 ± 0.9	810.3 ± 0.7	911.3 ± 0.9	239.4 ± 0.7	511.1 ± 0.6	1,162.3 ± 0.6	471.7 ± 0.4	504.7 ± 0.3

Lysine content of different sweet preserved hareer samples ranged from 910.1 to 922.5 mg/kg; moreover, the lysine content of sweet preserved hareer (control) is 923.43 mg/kg. The minimum value of leucine content has been found in sample S1L5, while the maximum value was exhibited in S2L2. Methionine content of different sweet preserved hareer samples ranged from 240.2 to 250.5 mg/kg; moreover, the methionine content of sweet preserved hareer (control) is 251.43 mg/kg. The minimum value of methionine content has been found in sample S3L5, while the maximum value was exhibited in S2L5. Phenylalanine content of different sweet preserved hareer samples ranged from 508.2 to 518.2 mg/kg; moreover, phenylalanine content of sweet preserved hareer (control) is 520.53 mg/kg. The minimum value of phenylalanine content has been found in sample S1L3, whereas the maximum value was exhibited in S2L1. Proline content of different sweet preserved hareer samples ranged from 1,160.5 to 1,172.6 mg/kg; moreover, the proline content of sweet preserved hareer (control) is 1,173.13 mg/kg. The minimum value of proline content has been found in sample S3L3, while the maximum value was exhibited in S2L2. Threonine content of different sweet preserved hareer samples ranged from 466.9 to 476.3 mg/kg; moreover, the threonine content of sweet preserved hareer (control) is 478.2 mg/kg. The minimum value of threonine content has been found in sample S1L5, while the maximum value was exhibited in S2L1. The valine content of different sweet preserved hareer samples ranged from 502.56 to 513.4 mg/kg; moreover, the valine content of sweet preserved hareer (control) is 514.8 mg/kg. The minimum value of valine content has been found in sample S1L4, while the maximum value was exhibited in S2L5 (Table 6).

**TABLE 6:** Nonessential amino acid profile of sweet preserved hareer

Brand	Cities	Alanine mg/kg	Arginine mg/kg	Aspartic acid mg/kg	Cysteine mg/kg	Glutamic acid mg/kg	Serine mg/kg	Tyrosine mg/kg	Glycine mg/kg
Control		628.8 ± 0.5	1,225.5 ± 0.7	7,259.7 ± 0.5	ND	1,574.2 ± 0.6	649.2 ± 0.7	631.3 ± 0.75	724.2 ± 0.6
S_1_	L_1_	618.2 ± 0.5	1,215.8 ± 0.6	7,249.3 ± 0.5	ND	1,567.2 ± 0.6	639.4 ± 0.7	625.56 ± 0.8	718.3 ± 0.6
	L_2_	616.3 ± 0.8	1,213.6 ± 0.5	7,247.2 ± 0.5	ND	1,564.833 ± 0.6	642.5333 ± 0.8	623.3 ± 0.8	713.3 ± 0.5
	L^3^	620.5 ± 0.75	1,212.3 ± 0.6	7,245.2 ± 0.4	ND	1,562.7 ± 0.5	637.3333 ± 0.8	621.4 ± 0.6	716.7 ± 0.6
	L_4_	621.5 ± 0.7	1,217.3 ± 0.6	7,251.6 ± 0.5	ND	1,561.267 ± 0.6	638.3667 ± 0.7	620.27 ± 0.7	717.9 ± 0.5
	L_5_	617.2 ± 0.7	1,216.3 ± 0.5	7,250.2 ± 0.5	ND	1,563.9 ± 0.7	639.4 ± 1.2	618.4 ± 0.7	714.8 ± 0.5
S_2_	L_1_	627.5 ± 0.6	1,224.2 ± 0.6	7,258.8 ± 0.6	ND	1,575.2 ± 0.5	648.9 ± 1.2	629.4 ± 0.7	723.7 ± 0.5
	L_2_	625.3 ± 0.5	1,222.3 ± 0.5	7,254.1 ± 0.4	ND	1,573.9 ± 0.5	646.3 ± 0.6	626.7 ± 0.3	721.8 ± 0.5
	L^3^	623.4 ± 0.7	1,221.8 ± 0.6	7,257.3 ± 0.5	ND	1,571.7 ± 0.5	644.4 ± 0.8	628.6 ± 0.9	719.2 ± 0.5
	L_4_	628.2 ± 0.6	1,223.3 ± 0.6	7,255.7 ± 0.4	ND	1,569.2 ± 0.5	645.6 ± 0.4	630.4 ± 0.6	718.2 ± 0.6
	L_5_	623.4 ± 0.5	1,225.9 ± 0.5	7,254.8 ± 0.5	ND	1,570.3 ± 0.6	643.4 ± 0.9	625.3 ± 0.8	721.8 ± 0.6
S_3_	L_1_	618.3 ± 0.6	1,219.6 ± 0.5	7,252.2 ± 0.6	ND	1,568.2 ± 0.6	643.4 ± 0.8	620.8 ± 0.7	717.7 ± 0.5
	L_2_	619.6 ± 0.5	1,216.8 ± 0.5	7,254.2 ± 0.5	ND	1,566.8 ± 0.5	639.3 ± 1	625.5 ± 1.15	713.5 ± 0.6
	L^3^	615.8 ± 0.5	1,215.9 ± 0.6	7,247.1 ± 0.8	ND	1,563.2 ± 0.6	637.4 ± 0.9	623.1 ± 0.7	718.6 ± 0.5
	L_4_	614.7 ± 0.5	1,214.5 ± 0.7	7,249.7 ± 0.6	ND	1,564.8 ± 0.6	639.3 ± 0.7	626.6 ± 0.5	714.7 ± 0.6
	L_5_	617.4 ± 0.5	1,217.7 ± 0.5	7,248.6 ± 0.6	ND	1,562.6 ± 0.5	640.5 ± 0.7	621.2 ± 0.9	715.2 ± 0.65
S_4_	L_1_	612.7 ± 0.5	1,218.6 ± 0.5	7,245.2 ± 0.4	ND	1,569.8 ± 0.9	634.8 ± 0.9	626.0 ± 0.2	716.7 ± 0.9
	L_2_	616.3 ± 0.5	1,214.3 ± 0.8	7,246.1 ± 0.8	ND	1,565.0 ± 0.2	637.1 ± 0.7	623.5 ± 0.6	713.8 ± 0.6
	L^3^	618.8 ± 0.4	1,218.5 ± 0.2	7,248.5 ± 0.2	ND	1,562.2 ± 0.7	639.2 ± 0.4	627.3 ± 0.7	718.7 ± 0.4
	L_4_	619.2 ± 0.7	1,212.4 ± 0.9	7,251.3 ± 0.9	ND	1,564.1 ± 1.1	641.9 ± 0.7	620.3 ± 0.9	712.8 ± 0.9
	L_5_	615.8 ± 0.6	1,214.7 ± 0.4	7,250.8 ± 0.1	ND	1,567.7 ± 0.6	640.9 ± 0.1	622.5 ± 1.1	714.3 ± 0.5

#### 3.2.4 Nonessential amino acid

Results showed that alanine content of different sweet preserved hareer samples ranged from 612.7 to 628.2 mg/kg; furthermore, the alanine content of sweet preserved hareer (control) is 628.8 mg/kg. The minimum value of alanine content has been found in sample S4L1, while the maximum value was exhibited in S2L4. Arginine content of different sweet preserved hareer samples ranged from 1,212.3 to 1,225.9 mg/kg; moreover, the arginine content of sweet preserved hareer (control) is 1,225.5 mg/kg. The minimum value of arginine content has been found in sample S1L3, while the maximum value was exhibited in S2L5. The aspartic acid content of different sweet preserved hareer samples ranged from 7,245.2 to 7,258.8 mg/kg; moreover, the aspartic acid content of sweet preserved hareer (control) is 7,259.7 mg/kg. The minimum value of arginine content has been found in sample S1L3, while the maximum value was exhibited in S2L1. Cysteine content in all the samples of sweet preserved hareer is nil. The glutamic acid content of different sweet preserved hareer samples ranged from 1,561.2 to 1,575.2 mg/kg; moreover, the glutamic acid content of sweet preserved hareer (control) is 1,574.2 mg/kg. The minimum value of glutamic acid content has been found in sample S1L4, while the maximum value was exhibited in S2L1.

The serine content of different sweet preserved hareer samples ranged from 634.8 to 648.9 mg/kg; moreover, the serine content of sweet preserved hareer (control) is 649.2 mg/kg. The minimum value of serine content has been found in sample S4L1, while the maximum value was exhibited in S2L1. Tyrosine content of different sweet preserved hareer samples ranged from 618.4 to 630.4 mg/kg; moreover, the tyrosine content of sweet preserved hareer (control) is 631.3 mg/kg. The minimum value of tyrosine content has been found in sample S1L5, while the maximum value was exhibited in S2L4. Glycine content of different sweet preserved hareer samples ranged from 712.8 to 723.7 mg/kg; moreover, the glycine content of sweet preserved hareer (control) is 724.2 mg/kg. The minimum value of glycine content has been found in sample S4L4, while the maximum value was exhibited in S2L1; Barthakur and Arnold (1991) also observed similar results.

## 4 CONCLUSION

The outcomes of the current scientific intervention strongly recommend that sample S2 taken from all the locations showed maximum amino acid and mineral contents. Moreover, sample S2 showed the maximum vitamin C, moisture, ash, pH, color, and extractive values, whereas acidity, TSS, and total plate count were observed minimum. *Salmonella* and *E. coli* were observed nil in all the samples. This research has opened a new arena of research for other scientists to explore potential phytochemicals of nutraceutical importance from this commodity.

## CONFLICT OF INTEREST

No conflict of interest.

## Data Availability

The data that support the findings of this study are available on request from the corresponding author. The data are not publicly available due to privacy or ethical restrictions.
